The article "The Modeling Analysis and Effect of CHI3L1 and CD31-Marked Microvessel Density in the Occurrence and Development of Cervical Squamous Cell Carcinoma" was published in 2022. Journal: Comput Math Methods Med.

# The Modeling Analysis and Effect of CHI3L1 and CD31-Marked Microvessel Density in the Occurrence and Development of Cervical Squamous Cell Carcinoma

**DOI:** 10.1155/2022/3516335

**Published:** 2022-06-18

**Authors:** Yanzi Qin, Wenjun Zhao

**Affiliations:** ^1^Department of Pathology, The First Affiliated Hospital of Bengbu Medical College, Bengbu, 233000 Anhui, China; ^2^Department of Emergency Internal Medicine, The Third the People's Hospital of Bengbu, Bengbu, 233000 Anhui, China

## Abstract

**Background:**

Chitinase-3-like protein 1 (CHI3Ll) has been identified as a novel tumor marker in several cancers. The objective of this study was to detect the expression of Chitinase-3-like protein 1 (CHI3L1) and CD31-labeled microvessel density (MVD) in cervical squamous cell carcinoma (CSCC) and to assess its prognostic impact.

**Methods:**

Elivision™ plus immunohistochemical method was used to detect CHI3L1 expression and MVD in different cervical tissues. We analyzed the relationship between CHI3L1 and MVD in CSCC tissues and investigated the relationship between CHI3L1, MVD, and clinicopathological parameters. Univariate and multivariate survival analyses were performed to assess the impact on progression-free survival (PFS) and overall survival (OS).

**Results:**

The positive expression rate of CHI3L1 protein in CSCC tissues (69.9%, 72/103) was significantly higher than that in high-grade cervical intraepithelial lesions (53.3%, 32/60), low-grade cervical intraepithelial lesions (25%, 15/60), and normal cervical tissues (16.7%, 10/60). MVD values ranged from 6 to 64 in CSCC, and no microvascular formation was observed in normal cervical tissues, high-grade intraepithelial lesions, or low-grade intraepithelial lesions. The high expression of CHI3L1 and MVD was significantly correlated with the invasion depth, differentiation degree, vascular invasion, and lymph node metastasis of CSCC (all *P* < 0.05). In CSCC, the expression of MVD in the CHI3L1 high-expression group (41.35 ± 9.056) was significantly higher than that in the CHI3L1 low-expression group (23.26 ± 11.000, *P* < 0.05). On univariate Kaplan–Meier analysis, FIGO stage, tumor diameter, lymph node metastasis, vascular invasion, CHI3L1, and MVD of CSCC were related to the prognosis of PFS and OS (all *P* < 0.05); however, CHI3L1 and MVD were not independent prognostic factors.

**Conclusion:**

CHI3L1 may be involved in the progression of cervical cancer. Its high expression can promote neovascularization in the tumor microenvironment. CHI3L1 is a potential therapeutic target in the context of cervical cancer.

## 1. Introduction

Globally, cervical cancer is one of the most common cancers and among the most common causes of cancer-associated mortality in women. The incidence of cervical cancer is particularly high in underdeveloped settings [1]. An estimated 600000 women worldwide are diagnosed with cervical cancer every year, and more than half of these die of this disease [2]. The main reasons for the deterioration of cervical cancer are infiltration and metastasis, resulting in a poor prognosis. Finding possible molecular targets that lead to the incidence and progression of cervical cancer is therefore crucial for the treatment and evaluation of cervical cancer patients in the future. Cervical cancer includes squamous cell carcinoma and adenocarcinoma, among which cervical squamous cell carcinoma (CSCC) is the most important histological type.

The article "The Modeling Analysis and Effect of CHI3L1 and CD31-Marked Microvessel Density in the Occurrence and Development of Cervical Squamous Cell Carcinoma" was published in 2022. Journal: Comput Math Methods Med.

Chitinase-3-like protein 1 (CHI3L1, also known as YKL-40), is located on human chromosome 1q32 [3]. As an important growth factor for connective tissue cells, CHI3L1 has been shown to regulate vascular endothelial growth factor and angiogenesis [4], differentiation, and proliferation of cells [5], reregulate the extracellular matrix [5], and activate Akt to participate in the migration of vascular endothelial cells [5]. It has important roles in signaling [6], preventing apoptosis [7], promoting metastasis [8], and tumor progression [5, 9–12]. Studies have demonstrated the involvement of CHI3L1 in tumor angiogenesis [13] and the formation of angiogenic mimicry in cervical cancer [14].

In a hypoxic environment, malignant tumor cells secrete proangiogenic factors, which promote the migration of vascular endothelial cells and formation of new blood vessels. Microvessel development has the potential to create tumor vascular networks, deliver nutrients to tumors, and further infiltrate the surrounding matrix. Tumor occurrence and metastasis are both influenced by microvessel density (MVD) [15, 16]. Many studies have found that tumor microvessels are closely linked to clinical progression and prognosis in a variety of solid tumors and that the expression of endothelial cell markers can be utilized to quantify the formation of MVD in tumor tissue [17]. CD31, also known as platelet endothelial cell adhesion molecule-1 (PPECAM-1), as one of the specific markers of endothelial cells, is often used to count tumor microvessels in immunohistochemical experiments to evaluate tumor angiogenesis [18].

This study is aimed at detecting the expression of CHI3L1 and MVD in CSCC and at the same time clarifying the relationship between CHI3L1 and MVD and its impact on the progression and evolution of disease. Our findings may provide a combination of targeted molecular therapy for cervical cancer.

## 2. Materials and Methods

### 2.1. Patients and Specimens

Paraffin archived specimens of 103 cases of CSCC tissues, 120 cases of cervical intraepithelial lesions (60 cases of high-grade intraepithelial lesions and 60 cases of low-grade intraepithelial lesions), and 60 cases of normal cervical epithelial tissues were retrospectively selected from the First Affiliated Hospital of Bengbu Medical College from January to December 2014. The pathological results of all cases were jointly diagnosed by two experienced senior pathologists, and all cases had complete clinical and follow-up data. Patients with CSCC were followed up until December 2021 or had died. In CSCC patients, the age ranged from 31 to 72 years, and the median age was 49 years old, mean ± standard deviation (49.0 ± 8.906) years old; tumor diameter is as follows: <2 cm in 10 cases, ≥2 cm and <4 cm in 50 cases, and ≥4 cm in 43 cases. The general types were endogenous infiltration in 24 cases, external lettuce flower in 30 cases, ulcer in 21 cases, and superficial erosion in 28 cases. Depth of infiltration is as follows: <1/2 full layer 42 cases, ≥1/2 and<2/3 full layer 40 cases, and ≥2/3 full layer 21 cases; degree of differentiation is as follows: high differentiation in 9 cases, medium differentiation in 63 cases, and low differentiation in 31 cases; 27 cases had lymph node metastasis, and 76 cases had no lymph node metastasis. Vascular invasion is as follows: 68 cases were found to have tumor thrombus, and 35 cases were found to have no tumor thrombus. According to the 2018 International Federation of Gynecology and Obstetrics (FIGO) staging criteria [19], there are 3 cases of IA1, 3 cases of IA2, 23 cases of IB1, 11 cases of IB2, 10 cases of IB3, 16 cases of IIA1, 10 cases of IIA2, 1 case of IIIA, 16 cases of IIIC1, 7 cases of IIIC2, and 3 cases of IVA. For the convenience of data statistics, the cases in this study are divided into IA (IA1+IA2), IB (IB1+IB2+IB3), II (IIA1+IIA2), and III+IV (IIIA+IIIC1+IIIC2+IVA). All patients did not receive any radiotherapy or chemotherapy before surgery. The ethics committee of Bengbu Medical College has approved the implementation of this experiment.

The article "The Modeling Analysis and Effect of CHI3L1 and CD31-Marked Microvessel Density in the Occurrence and Development of Cervical Squamous Cell Carcinoma" was published in 2022. Journal: Comput Math Methods Med.

### 2.2. Immunohistochemistry

The collected cervical tissues were fixed with 10% neutral formalin, paraffin-embedded, and sequentially sectioned (3~5 *μ*m thick sections). Tissue antigens were restored after deparaffinization and hydration of paraffin slices. Phosphate-buffered solution (PBS) was diluted three times to eliminate the PBS solution. Diluted with 50 *μ*l of primary antibody per section (CHI3L1, rabbit polyclonal, diluted 1 : 1000, Abcam, USA and CD31, rabbit polyclonal, diluted 1 : 200, Abcam, USA), overnight at 4°C. Wash with PBS 3 times, remove PBS solution, add 50 *μ*l polymer reinforcement to each section, incubate at room temperature for 20 min, and rinse with PBS 3 times. Remove PBS solution, add 50 *μ*l enzyme-labeled anti-mouse/rabbit polymer (secondary antibody) to each section, and incubate at room temperature for 30 min. Rinse with PBS 3 times. The slices were stained with DAB (3,3′-diaminobenzidine) and observed under a microlens for 3~5 minutes. Hematoxylin was restained and turned blue with PBS. PBS replaced primary antibodies as negative control and known positive tablets as a positive control. The above experiments were performed according to the Elivision™ Plus detection kit instructions (Fuzhou Maixin Co., Ltd., China).

### 2.3. Positive Criteria for CHI3L1

CHI3L1 positive particles are light yellow to brownish yellow, mainly located in the cytoplasm. Immunohistochemical labeling results were evaluated by the semiquantitative scoring method from staining intensity and staining range. We randomly selected five high-power fields (400x) in the tumor cell region, and 200 tumor cells were counted. According to the proportion of positive cells, the cells were divided into <5% as 0, 5%-~25% as 1, 26%~50% as 1, 51%~75% as 3, and >75% as 4. Staining intensity of positive cells is as follows: no staining as 0, light yellow as 1, brown-yellow as 2, and tan as 3. When the two of the same case are multiplied, the standard of low expression or no expression is <3 points and the standard of high expression is ≥3. All results were judged by the double-blind method and repeated three times.

### 2.4. MVD Positive Evaluation Criteria

MVD was counted by Weinner counting method [20]. At low magnification (100x), the area with the highest microvascular density was selected. At medium magnification (200x), the number of microvessels in 5 different fields was manually counted and the average value was MVD. CD31 was located in vascular endothelial cells, and a positive microvessel was counted as a single endothelial cell or endothelial cell cluster with positive staining. Inclusion criteria are as follows: endothelial cells with complete structural outline were stained, isolated from adjacent microvessels showed single vascular endothelial cells or clusters of vascular endothelial cells and branching vascular structures with unconnected structures. Exclusion criteria are as follows: vessels with diameter ≥ 8 red blood cells, thick-walled smooth muscle vessels, and vessels in the sclerotic necrotic zone. All of the results were judged three times using the double-blind approach.

### 2.5. Statistical Analysis

All data were collected by SPSS26.0 (IBM Corp., Armonk, NY, USA) statistical software analysis. Statistically, the cut-off value is 0.05. When *P* < 0.05, it was statistically significant. *t*-test or Fisher's exact test was used for measurement data of both groups, one-way ANOVA was used for measurement data of multiple groups, and *χ*^2^ test was used for counting data. The follow-up data were analyzed by the Kaplan–Meier method for univariate survival and Cox regression analysis for multivariate survival.

The article "The Modeling Analysis and Effect of CHI3L1 and CD31-Marked Microvessel Density in the Occurrence and Development of Cervical Squamous Cell Carcinoma" was published in 2022. Journal: Comput Math Methods Med.

## 3. Result

In this section, we explain the expression of CHI3L1 in different cervical tissues, the relationship between the expression of CHI3L1 in CSCC tissues and its clinical parameters in patients, and the expression of CD31-marked MVD in different cervical tissues in detail.

### 3.1. Expression of CHI3L1 in Different Cervical Tissues

The positive expression rate of CHI3L1 was 16.7% (10/60), 25% (15/60), 53.3% (32/60), and 69.9% (72/103) in normal cervical tissues, low-grade intraepithelial lesions, high-grade intraepithelial lesions, and CSCC, respectively. The positive expression of CHI3L1 in cervical tissues increased during the progression of malignant transformation (*χ*^2^ = 56.486, *P* < 0.001), which was statistically significant. Meanwhile, the positive expression rate of CHI3L1 in CSCC tissues was significantly higher than that in normal cervical tissues, low-grade intraepithelial lesions, and high-grade intraepithelial lesions (*χ*^2^ = 42.983, *χ*^2^ = 30.718, and *χ*^2^ = 4.507, all *P* < 0.05). The positive expression of CHI3L1 in high-grade intraepithelial lesions was significantly higher than that in normal cervical tissues and low-grade intraepithelial lesions (*χ*^2^ = 17.729 and *χ*^2^ = 10.108, both *P* < 0.05). However, there was no significant difference in the positive expression of CHI3L1 between low-grade intraepithelial lesions and normal cervical tissue, as shown in Figure 1.

### 3.2. The Relationship between the Expression of CHI3L1 in CSCC Tissues and Its Clinical Parameters of Patients

The results showed that in CSCC tissues, the positive expression rate of CHI3L1 was significantly correlated with the depth of tumor invasion, degree of differentiation, vascular invasion, and lymph node metastasis (all *P* < 0.05), but not with the patient's age, tumor diameter, gross type, and FIGO stage (all *P* > 0.05). With the deepening of tumor infiltration, especially the infiltration depth of more than 2/3 of the full thickness, the positive rate of CHI3L1 (85.7%, 18/21) was significantly higher than that of the infiltration depth of less than 1/2 of the full thickness (50%, 21/42) and the positive rate of more than 1/2 but less than 2/3 full-thickness (82.5%, 33/40). The positive rate of CHI3L1 in poorly differentiated tissues (96.7%, 30/31) was significantly higher than that in well-differentiated tissues (11.1%, 1/9) and moderately differentiated tissues (65.1%, 41/63). The CHI3L1 protein-positive rate in patients with lymph node metastasis (85.2%, 23/27) was significantly higher than that in patients without lymph node metastasis (64.5%, 49/76). The positive rate (88.2%, 60/68) was higher than the positive rate of patients without intravascular tumor thrombus (34.3%, 12/35). The above data are shown in Table 1.

The article "The Modeling Analysis and Effect of CHI3L1 and CD31-Marked Microvessel Density in the Occurrence and Development of Cervical Squamous Cell Carcinoma" was published in 2022. Journal: Comput Math Methods Med.

### 3.3. Expression of CD31-Marked MVD in Different Cervical Tissues

In 103 cases of CSCC tissues, MVD was mainly characterized by irregular morphology, increased number, and disorganized branching and was concentrated at the edge of tumor invasion. MVD values ranged from 6 to 64, with the median value of 36 as the truncated value. MVD in the high-expression group was ≥36, and MVD in the low-expression group was <36, as shown in Figures 1(e) and 1(f). No microvascular formation was detected in normal cervical tissues, low-grade intraepithelial lesions, and high-grade intraepithelial lesions, and only CD31-marked MVD was detected in CSCC tissues, suggesting that the production of MVD generation increased significantly after cervical tissue carcinogenesis.

### 3.4. The Relationship between the Expression of MVD in CSCC Tissues and Its Clinicopathological Parameters

Further analysis showed that MVD expression in CSCC tissues was correlated with tumor size, invasion depth, differentiation type, vascular invasion, and lymph node metastasis (*P* < 0.05), but not with age, tumor gross type, and FIGO stage (*P* > 0.05). With the increase in tumor diameter, the MVD value increased gradually (*F* = 10.123, *P* < 0.05). The MVD value of cases with invasion depth of tumor invasion was 1/2 of the full layer (≥2/3 full layer, 38.90 ± 11.458 and ≥1/2 and<2/3 full layer, 39.15 ± 11.116) was significantly higher than that of cases with invasion depth of <1/2 full layer (31.31 ± 13.616). The more poorly differentiated the tumor was, the higher the MVD value was (*F* = 12.151, *P* < 0.05). The MVD value of the CSCC patients with lymph node metastasis (44.70 ± 9.376) was significantly higher than that of patients without lymph node metastasis (32.78 ± 12.341). The MVD value of CSCC with vascular invasion (41.56 ± 9.670) was significantly higher than that of CSCC without vascular invasion (24.91 ± 10.678). The above data are shown in Table 1.

### 3.5. The Relationship between CHI3L1 and MVD in CSCC Tissue

CSCC tissues were divided into two groups: the high CHI3L1 expression group and the low CHI3L1 expression group. MVD value of the high-expression group of CHI3L1 was 41.83 ± 10.024, while that of the low-expression group of CHI3L1 was 23.03 ± 11.020, and the difference was statistically significant (*t* = 8.473, *P* < 0.05). The positive rate of MVD in the group with high CHI3L1 expression was higher than that in the group with low CHI3L1 expression, as shown in Table 2.

The article "The Modeling Analysis and Effect of CHI3L1 and CD31-Marked Microvessel Density in the Occurrence and Development of Cervical Squamous Cell Carcinoma" was published in 2022. Journal: Comput Math Methods Med.

### 3.6. Prognosis

The overall survival (OS) and progression-free survival (PFS) after operation in 103 patients were evaluated to see if there was a link between the expression of CHI3L1 and MVD in CSCC and patient survival. Kaplan–Meier (log-rank) survival analysis was performed on the relevant data. The results showed that the OS survival time of CSCC patients over five years after operation was 82.42 ± 15.789 months, and the OS survival rate over five years was 66.9% (69/103). The survival time of PFS was 74.63 ± 21.630 months, and the survival rate of PFS over five years was 50.4% (52/103). FIGO stage (log − rank = 26.469, *P* < 0.001), tumor diameter (log − rank = 8.779, *P* = 0.012), depth of invasion (log − rank = 6.108, *P* = 0.047), degree of differentiation (log − rank = 7.689, *P* = 0.021), lymph node metastasis (log − rank = 33.316, *P* < 0.001), vascular invasion (log − rank = 17.062, *P* < 0.001), CHI3L1 expression (log − rank = 12.655, *P* < 0.001, Figure 2(a)), and MVD expression (log − rank = 7.248, *P* = 0.007, Figure 2(b)) correlated with OS prognosis (*P* < 0.05). FIGO stage (log − rank = 13.084, *P* < 0.001), tumor diameter (log − rank = 14.211, *P* = 0.001), depth of invasion (log − rank = 6.108, *P* = 0.047), degree of differentiation (log − rank = 13.084, *P* = 0.001), lymph node metastasis (log − rank = 39.522, *P* < 0.001), vascular invasion (log − rank = 25.180, *P* < 0.001), CHI3L1 expression (log − rank = 24.431, *P* < 0.001, as shown in Figure 2(c)), and MVD expression (log − rank = 8.522, *P* = 0.004, as shown in Figure 2(d)) were correlated with PFS prognosis (*P* < 0.05). Cox multivariate analysis is shown in Tables 3 and 4.

## 4. Discussion and Conclusion

CHI3L1 can be expressed and secreted by a variety of cells, including macrophages, neutrophils, epithelial cells, smooth muscle cells, chondrocytes, and tumor cells [21]. In recent years, more and more investigations on CHI3L1 in malignant tumors have been conducted. Serum CHI3L1 levels are significantly increased in endometrial cancer, melanoma, colorectal cancer, lung cancer, and breast cancer [22–24]. Increased serum CHI3L1 protein level in patients with CSCC and cervical adenocarcinoma was shown to lead to aggravation of cervical cancer, resulting in poorer prognosis and shorter survival [25, 26]. The expression level of CHI3L1 protein in cervical cancer tissues was also shown to be significantly higher than that in normal cervical tissues [13]. Although several studies have demonstrated the involvement of high expression of serum CHI3L1 protein in the growth, proliferation, infiltration, and metastasis of cervical cancer [21, 25, 26], the relationship between the expression level of CHI3L1 protein and the specific clinicopathological parameters of cervical cancer patients from the perspective of histology is not well characterized. Only Ngernyuang et al. [13] reported a much higher positivity rate of CHI3L1 in cervical cancer patients with regional lymph node and organ metastasis compared to that in patients with nonmetastatic disease, which is consistent with the results of the present study. In the present study, we detected the expression level of CHI3L1 in different cervical tissue samples and confirmed that the positive expression rate of CHI3L1 in CSCC tissues was significantly higher than that in cervical intraepithelial lesions and normal cervical tissues, which was consistent with the results reported above [13]. The presence of lymph node metastases in CSCC patients enhanced the expression level of the CHI3L1 protein, according to this study (*P* < 0.05). Meanwhile, it was confirmed for the first time in this study that the protein level of CHI3L1 was significantly increased with the lower differentiation degree of CSCC, the deepening of tumor invasion depth or vascular invasion (all *P* < 0.05). These findings suggest that dynamic monitoring of the positive expression level of CHI3L1 in cervical tissue may predict whether the cervix will undergo malignant changes, so CHI3L1 may become a candidate gene for predicting cervical cancer. The high expression of CHI3L1 protein is closely related to lymph node metastasis and tumor invasion of cervical cancer, which may aggravate the progression of cervical cancer.

The article "The Modeling Analysis and Effect of CHI3L1 and CD31-Marked Microvessel Density in the Occurrence and Development of Cervical Squamous Cell Carcinoma" was published in 2022. Journal: Comput Math Methods Med.

How does CHI3L1 participate in the occurrence and progression of cervical cancer, and what is the specific mechanism? One of the leading causes of death in cancer patients is tumor metastasis and dissemination. Microangiogenesis and dietary factors are primarily used by lymph node metastases and hematogenous dissemination to offer ample blood supply. Tumor metastasis and spread are one of the causes of death in cancer patients. Lymph node metastasis and hematogenous dissemination mainly rely on microangiogenesis to provide abundant blood supply and nutritional factors. Growth and migration cannot leave the blood vessels that provide nutrients and energy. In order to ensure the survival and growth of malignant tumor cells, a continuous blood supply is required, and a good blood supply can further maintain and promote the growth of malignant tumor cells. Genogenesis plays an extremely important role in the occurrence and development of tumor tissues [27]. It has been reported that CHI3L1 plays a key role in tumor development by promoting tumor angiogenesis [6, 28]. Based on this, the relationship between MVD and clinicopathological parameters of CSCC and CHI3L1 was also detected in this study. No microvascular formation was observed in the control tissues (cervical intraepithelial lesions and normal cervical tissues), while a higher number of MVD was observed in cervical tissues, which is consistent with previous reports [13]. This experiment showed that the number of MVD would increase with the increase of tumor, the deepening of invasion depth, the lower degree of differentiation, lymph node metastasis, and vascular invasion, suggesting that the occurrence and deterioration of CSCC are closely related to the formation of neovascularization.

This study was the first to explore the effects of CHI3L1 and MVD on the prognosis and survival of CSCC from the histological perspective. The study showed that the survival status of OS and PFS was related to the expression of CHI3L1 protein and MVD (*P* < 0.05). However, CHI3L1 expression cannot be used as an independent prognostic factor for OS and DFS in CSCC patients, nor can MVD expression be used as an independent prognostic factor for OS in CSCC patients, while MVD expression level can be used as an independent factor to evaluate the survival of PFS. It is suggested that high expression of CHI3L1 protein and MVD may indicate poor prognosis of CSCC patients, but neither of them can be used as independent prognostic criteria for CSCC. A similar conclusion was obtained in detecting the influence of serum CHI3L1 expression level on the prognosis of cervical cancer [25]. Mitsuhashi et al. [25] showed in a retrospective study that high serum CHI3L1 protein level is a potential independent prognostic biomarker for assessing short-term OS before treatment in patients with CSCC and cervical adenocarcinoma. This study also confirmed that FIGO stage, tumor size, lymph node metastasis, and vascular invasion were correlated with the prognosis of OS and PFS in patients with ESCC (*P* < 0.05), and these factors were key factors affecting the prognosis of patients.

In this study, the number of MVD in the high-expression group of CHI3L1 was significantly higher than that in the low-expression group of CHI3L1, suggesting that CHI3L1 may be involved in the occurrence and development of cervical cancer and promote tumor angiogenesis as an angiogenic factor. Ngernyuang et al. [13] also reached the same conclusion in previous studies. Studies have shown that CHI3L1 is involved in the adhesion and migration of vascular endothelial cells [4, 29]. Studies have shown that the addition of CHI3L1 recombinant protein in vitro promotes vascular endothelial cell migration and tubule formation, which are important steps in angiogenesis. Moreover, CHI3L1 can promote the secretion of vascular endothelial growth factor (VEGF) by U87 cells and accelerate tumor angiogenesis by cooperating with other proangiogenic factors [4]. CHI3L1 activates the activities of focal adhesion kinase (FAK) and extracellular regulated protein kinase (ex-tracellular signal regulated kinases-1, ERK-1)/(ex-tracellular signaI regulated kinases-2, ERK-2). Increased VEGF and angiogenesis [30], in particular the membrane receptor syndeca-1 and integrin *α*v*β*5, act as triggering molecules to trigger the CHI3L1 signaling cascade. CHI3L1 binds to the receptor of advanced dycation endproducts (RAGE) and induces the proliferation of cancer cells. ERK1/2-MAPK (mitogen activated protein kinase) pathway plays a role in the downstream signal cascade of RAGE-CHI3L1 [30]. Therefore, the next step of this research group is to detect the relationship between CHI3L1 and MVD through in vitro experiments, to further analyze the role of CHI3L1 in the formation of new blood vessels in CSCC and to explore the mechanism of CHI3L1 involved in CSCC.

The article "The Modeling Analysis and Effect of CHI3L1 and CD31-Marked Microvessel Density in the Occurrence and Development of Cervical Squamous Cell Carcinoma" was published in 2022. Journal: Comput Math Methods Med.

In general, the tumor size, FIGO stage, invasion depth, vascular invasion, lymph node metastasis, and differentiation degree of CSCC are all linked to high CHI3L1 and MVD expression. The high expression of CHI3L1 and MVD may indicate a poor prognosis for patients, but it cannot be used as an independent prognostic factor to evaluate the prognosis of patients with cervical cancer. Studies have pointed out that the growth and progression of tumors can be effectively controlled by controlling tumor angiogenesis [31]. It seems plausible that targeted inhibition of CHI3L1 expression level may potentially control tumor neovascularization and inhibit generation of lymphatic vessels, so as to effectively control tumor growth and progression.

## Figures and Tables

**Figure 1:** Immunohistochemical analysis of CHI3L1 and MVD expression in cervical squamous cell carcinoma (CSCC) and control groups (×400 magnification). CHI3L1 was negatively expressed in (a) normal cervical tissue. CHI3L1 (red arrow) is brown or tan granules in the cytoplasm in (b) low-grade intraepithelial lesions, (c) high-grade intraepithelial lesions, and (d) ESCC, respectively. CD31-marked microvessels are expressed between nests of (e, f, black arrows) ESCC.

The article "The Modeling Analysis and Effect of CHI3L1 and CD31-Marked Microvessel Density in the Occurrence and Development of Cervical Squamous Cell Carcinoma" was published in 2022. Journal: Comput Math Methods Med.

**Figure 2:** Kaplan–Meier analysis of the survival rates of patients with CSCC: (a) lower overall survival (OS) of patients with positive CHI3L1 expression (log − rank = 12.655, *P* < 0.001), (b) lower OS of patients with positive MVD expression (log − rank = 7.248, *P* = 0.007), (c) progression-free survival (PFS) of patients in relation to CHI3L1 (log − rank = 24.431, *P* < 0.001), and (d) lower PFS of patients with positive MVD expression (log − rank = 8.522, *P* = 0.004).

**Table 1:** The relationship between CHI3L1, MVD, and clinicopathological parameters of cervical squamous cell carcinoma (CSCC).

Variable	CHI3L1		*χ* ^2^	*P*	MVD	*t*-test/ANOVA	*P*
	High expression	Low expression					
Age (years)			2.356	0.125		7.985	0.357
<50	37	21			34.88 ± 12.802		
≥50	35	10			37.22 ± 12.669		
Diameter (cm)			1.785	0.410		10.123	0.001
<2	6	4			20.60 ± 10.255		
≥2, <4	33	17			35.98 ± 11.531		
≥4	33	10			39.12 ± 12.204		
General type			2.522	0.471		2.068	0.109
Endogenous infiltration	15	9			34.38 ± 14.080		
External lettuce flower	24	6			38.57 ± 11.726		
Ulcer	15	6			39.29 ± 10.494		
Superficial erosion	18	10			31.82 ± 13.358		
Depth of infiltration			13.420	0.001		4.975	0.009
<1/2	21	21			31.31 ± 13.616		
≥1/2, 2/3	33	7			39.15 ± 11.116		
≥2/3	18	3			38.90 ± 11.458		
Differentiation			26.122	0.001		12.151	0.001
Well	1	8			21.44 ± 13.602		
Moderately	41	22			34.81 ± 12.076		
Poorly	30	1			42.32 ± 9.639		
Lymph node metastasis			4.062	0.044		4.570	0.001
Yes	23	4			44.70 ± 9.376		
No	49	27			32.78 ± 12.341		
Vascular invasion			31.967	0.001		7.985	0.001
Yes	60	8			41.56 ± 9.670		
No	12	23			24.91 ± 10.678		
FIGO stage			2.296	0.513		1.591	0.196
IA	3	3			26.17 ± 15.690		
IB	29	15			35.36 ± 11.654		
II	20	6			38.46 ± 11.863		
III+IV	20	7			36.48 ± 14.132		

**Table 2:** The relationship between CHI3L1 and MVD in CSCC.

Variable	MVD	*t*	*P*
CHI3L1		8.473	0.001
High expression	41.83 ± 10.024		
Low expression	23.03 ± 11.020		

**Table 3:** Results of multivariate Cox regression analysis of overall survival (OS).

	*B*	SE	Wald	df	*P*	Exp (*B*)	95.0% CI for Exp (*B*)	
							Lower	Upper
Age (years)	0.505	0.384	1.732	1	0.188	1.657	0.781	3.514
FIGO stage	-0.817	0.545	2.250	1	0.134	0.442	0.152	1.285
Diameter (cm)	0.551	0.392	1.972	1	0.160	1.735	0.804	3.745
Depth of infiltration	-0.282	0.286	.973	1	0.324	0.754	0.431	1.321
Differentiated	0.433	0.396	1.197	1	0.274	1.542	0.710	3.352
Lymph node metastasis	-2.618	1.075	5.927	1	0.015	0.073	0.009	0.600
General type	-0.456	0.325	1.970	1	0.160	0.634	0.335	1.198
Vascular invasion	-0.946	0.886	1.140	1	0.286	0.388	0.068	2.204
CHI3L1	-1.219	0.816	2.232	1	0.135	0.296	0.060	1.463
MVD	0.587	0.446	1.731	1	0.188	1.798	0.750	4.312

The article "The Modeling Analysis and Effect of CHI3L1 and CD31-Marked Microvessel Density in the Occurrence and Development of Cervical Squamous Cell Carcinoma" was published in 2022. Journal: Comput Math Methods Med.

**Table 4:** Results of multivariate Cox regression analysis of progression-free survival (PFS).

	*B*	SE	Wald	df	*P*	Exp (*B*)	95.0% CI for Exp (*B*)	
							Lower	Upper
Age (years)	0.130	0.313	0.171	1	0.679	1.138	0.616	2.103
FIGO stage	-0.387	0.415	0.867	1	0.352	0.679	0.301	1.533
Diameter (cm)	0.592	0.308	3.691	1	0.055	1.808	0.988	3.307
Depth of infiltration	-0.365	0.233	2.454	1	0.117	0.694	0.440	1.096
Differentiated	0.401	0.337	1.414	1	0.234	1.494	0.771	2.893
Lymph node metastasis	-1.792	0.807	4.931	1	0.026	0.167	0.034	0.810
General type	-0.618	0.273	5.123	1	0.024	0.539	0.316	0.921
Vascular invasion	-0.564	0.608	0.859	1	0.354	0.569	0.173	1.875
CHI3L1	-1.867	0.676	7.617	1	0.006	0.155	0.041	0.582
MVD	0.502	0.357	1.972	1	0.160	1.652	0.820	3.328

## Data Availability

All data generated or analyzed during this study are included in this published article.
